# In‐hospital outcomes of patients with a hypertensive emergency at a medical center, Ethiopia: A prospective observational study

**DOI:** 10.1002/hsr2.845

**Published:** 2022-09-22

**Authors:** Mengist Awoke Yizengaw, Kisi Chemeda, Kabaye Kumela, Behailu Terefe Tesfaye

**Affiliations:** ^1^ Department of Clinical Pharmacy, School of Pharmacy, Institute of Health Jimma University Jimma Ethiopia; ^2^ Department of Pharmacy Jimma Medical Center Jimma Ethiopia

**Keywords:** emergency, Ethiopia, high blood pressure, mortality, outcome health care

## Abstract

**Background:**

Hypertensive emergency is associated with substantial complications and loss of life across the world. Early identification and treatment of hypertensive emergency complications are critical to prevent or avoid any consequences. Despite this, in Ethiopia, studies addressing mortality rate and its predictors as well as complications of hypertensive emergency are limited.

**Aims:**

This study aim to evaluate in‐hospital mortality of patients admitted with a hypertensive emergency at the emergency ward of Jimma Medical Center.

**Methods:**

A consecutive sample of 140 adult (≥18 years of age) patients with a hypertensive emergency were recruited from September 1, 2020 to February 25, 2021 at Jimma Medical Center, Ethiopia and were followed up from admission to discharge/death. Patients who declined to participate and readmitted during the study period were excluded. To assess factors associated with in‐hospital mortality, bivariate and multivariate Cox regression analyses were performed. A *p* value of less than 0.05 was used to declare the statistical significance.

**Results:**

Over three‐fourths of the study participants, that is, 108 (77.1%), were males with a mean (±standard deviation) age of 52.8 ± 13.6 years. Hemorrhagic stroke, 53 (38.0%), and acute kidney injury, 38 (27.1%), were the most common complications of hypertensive emergency. The average (±standard deviation) length of stay in the hospital was 8.53 ± 3.61 days. During in‐hospital follow‐up, 16 patients (11.4%, 95% confidence interval: 6.7–17.9) died. Multivariate Cox regression analysis showed that there was a significant relationship between patients not doing regular physical exercise before the current admission (adjusted hazard ratio = 4.629, 95% confidence interval: 1.171–18.294, *p* = 0.015) and in‐hospital mortality.

**Conclusion:**

More than one‐tenth of patients with hypertensive emergency death was recorded at Jimma Medical Center. The frequent complications of hypertensive emergency were hemorrhagic stroke and acute renal injury. Not doing regular physical exercise before the current admission raises the likelihood of in‐hospital death. Therefore, strengthening and encouraging patients to perform regular physical exercise is imperative.

## 1 BACKGROUND

Hypertensive emergency (HE) is a persistent elevation in systolic blood pressure (SBP) ≥ 180 mmHg and/or diastolic blood pressure (DBP) ≥ 110 mmHg with acute or ongoing target‐organ injury (TOI).^1^, ^2^ Hemorrhages, exudates, or papilledema of the eye, acute pulmonary edema, hypertensive encephalopathy, stroke, acute myocardial infarction, and acute renal failure are common examples of TOI.^3^, ^4^ The common risk factors for HE are obesity, uncontrolled hypertension, health comorbid conditions, sedentary lifestyle, polypharmacy, noncompliance to antihypertensive medications, and diet.^5^, ^6^, ^7^

Uncontrolled BP is the most common modifiable cause of mortality and disability across the world.^8^ Globally, uncontrolled BP was associated with approximately 8.5 million fatalities in 2015, with 88% of those deaths occurring in low‐ and middle‐income nations.^9^ The mortality from complicated hypertension is threefold higher in sub‐Saharan Africa (SSA),^10^ with the range of 11.6%^11^ to 42.9%^12^ of in‐hospital mortality among HE cases. Hypertension is the seventh most common reason for mortality in Ethiopia, representing 1.4% of all mortalities.^13^

Treatment for HE is decided based on clinical experience, insights, and intermediate result assessments. Patients presenting with HE requires immediate intervention, to avoid or reduce more hypertensive harm while preventing hypotension and associated consequences and mortalities.^1^ Although the optimal target for BP lowering in HE is still uncertain worldwide, personalized treatment is required depending on the nature and magnitude of damage, level of BP elevation, and in particular medication side effects on comorbid conditions.^6^, ^14^, ^15^, ^16^

To safely lower the elevated blood pressure, safeguard target organ function, increase symptoms, decrease complications, and enhance clinical outcomes, patients with HE require the administration of effective and fast‐acting intravenous medicines.^4^, ^17^ In these patient populations, the recommended intravenous medications and the target BP reduction vary based on the specific end‐organ damage.^4^, ^18^, ^19^, ^20^, ^21^

In Africa, including SSA, data on in‐hospital, as well as the long‐term, outcomes of HE are limited.^22^, ^23^ In Ethiopia, uncontrolled BP is increasing with an estimated pooled prevalence of 48% (95% confidence interval [CI]: 36–61)^24^ and it is as high as 57.2% at the Jimma Medical Center (JMC),^25^ which increases hypertensive‐related organ damages and mortality.^26^, ^27^ Despite an increment in the prevalence of uncontrolled BP in Ethiopia, only a few studies reported admission outcomes of HE.^11^, ^26^ Therefore, the primary aim of this study was to evaluate in‐hospital mortality and its associated factors of HE. Additionally, the study evaluated the clinical complications and duration of hospital stay of patients with HE at JMC, southwest Ethiopia.

## 2 METHODS

### 2.1 Study design and setting

A prospective facility‐based observational study was employed at the emergency and medical ward of JMC from September 1, 2020 to February 25, 2021; the only teaching and medical center in Southwest Ethiopia. It is 352 km far from Addis Ababa, the capital. It serves about 11,000 emergency cases per year, including hypertensive emergencies.

### 2.2 Populations

#### 2.2.1 Source populations

All adult patients hospitalized with HE at JMC's emergency ward.

#### 2.2.2 Study populations

All eligible adult patients hospitalized with HE at the emergency ward of JMC throughout the study duration.

### 2.3 Criteria for eligibility

#### 2.3.1 Inclusion criteria

- Age ≥ 18 years and diagnosed with HE.

#### 2.3.2 Exclusion criteria

- Patients readmitted during the study period.

### 2.4 Sample size determination and sampling technique

The size of the sample (*n*) was calculated by using single population proportion formula using the proportion (*p*) of in‐hospital mortality among hypertensive patients, with target organ damage in Addis Ababa, Ethiopia being 16.9% (*p* = 0.168),^26^ with a 95% CI, 5% margin of error, and adjusting for the finite admission of 300 HE patients to JMC's emergency unit in 2019. Adding 10% of the nonresponse rate, finally, 140 hospitalized adults with HE at JMC during the study perio who met the inclusion criteria were recruited. Study participants were formed using a consecutive sampling technique.

### 2.5 Instruments and procedures for data collection

After reviewing relevant literatures, the data collection tool was developed. Face‐to‐face interviews with patients and a review of their medical records were used to collect data. Four trained health professionals (two Bachelor's degree pharmacists and two Bachelor's degree nurses) were employed for the data collection. The data collection tools comprised sociodemographic‐related factors such as age, sex, residence, marital status, educational status, and occupations, behavioral related (self‐reported khat chewing, alcohol drinking, cigarette smoking status; physical exercise, salt consumption, and medication adherence), clinical characteristics and investigations (comorbidities, on admission clinical manifestations, types of hypertension diagnosis (newly/known), BP measurement on admission and at discharge/death, and medication‐related (antihypertensive medications used at inpatient setting) variables. Data on the duration of antihypertensive medication, previous antihypertensive medication, and potential reasons for discontinuing medication were collected through face‐to‐face interviews. Data on medical conditions were gathered from the patients' medical charts. While the patient was sitting, a mercury sphygmomanometer was used to take blood pressure at various intervals. An average BP measurement on the date of admission and discharge/death was recorded. Target‐organ damage/complications secondary to HE like ischemic/hemorrhagic stroke, dissection of the aorta, acute kidney injury, encephalopathy, ST‐elevated myocardial infarction (STEMI), acute congestive heart failure, and hypertensive retinopathy developed on admission or during their hospitalization were recorded from the patient chart.

The target organ damage was diagnosed by attending physicians according to the following findings. With the help of a noncontrast computed tomography (CT) or magnetic resonance imaging of the skull, ischemic/hemorrhagic stroke was defined as a fast‐growing clinical sign of localized (at times global) disruption of brain function lasting more than 24 h.^28^ Aortic dissection is defined as a situation in which the intima of the aortic wall has separated, as shown by a CT scan, allowing the flow of blood into an artificial route made up of the inner and outer layers of the media.^29^ Acute kidney injury is defined as a 0.3 mg/dl increase in serum creatinine in 48 h or a urine output of less than 0.5 ml/kg/h for 6 h.^30^ STEMI diagnosis is secured when troponin levels rise and/or fall, along with supporting evidence such as clinical manifestations, suggestive electrocardiographic variations, or new evidence of viable myocardial loss or a new regional wall motion anomaly on imaging.^31^ Hypertensive retinopathy was diagnosed based on retinal or fundus examination showing narrowing of blood vessels with/without an abnormal vascular permeability leading to retinal edema, flame‐shaped hemorrhages, and formation of hard exudates.^32^ Patients with high blood pressure, changed mental status, visual abnormalities, headaches, or seizures were considered as the diagnosis component of hypertensive encephalopathy, which is supported by a CT scan to discover brain abnormalities.^33^

### 2.6 Outcome variable

In‐hospital mortality from all causes, complications, factors associated with mortality, and length of stay at the hospital.

### 2.7 Outcome validation

The study participants were followed from the time of admission until their discharge/death, that is, emergency ward plus medical ward staying (if transferred to) period. All‐cause, in‐hospital mortality was recorded from the patient chart including time to death after admission. The time interval between the patient's entrance date and departure date from the hospital was used to calculate the length of hospital stay.

### 2.8 Assurance of data quality

To ensure consistency, the data abstraction tools were first written in English, thereafter translated into two commonly used local languages (Amharic and Afaan Oromo), and back‐translated into English by a third party. Before beginning the real data gathering, the tool was pretested, and the necessary adjustments were made. Before analysis, the data were assembled, coded, and checked for consistency.

### 2.9 Data processing and analysis

The data were entered into Epidata version 4.6.0.5 and afterwards exported to the Statistical Package for Social Science version 23.0 for analysis. The frequency and percentage were used to present the categorical data. A normality test was done for continuous data using the Shapiro–Wilk's *W*‐test. Then, the median and interquartile range (IQR) were used to report nonparametric data, whereas mean ± standard deviation was used to report parametric data. Cell adequacy was verified for all categorical data. The Kaplan–Meier survival analysis of mortality was conducted using the time frame from admission to discharge/death and whether or not regular physical exercise was done as independent factors. To compare in‐hospital survival, the log‐rank test was used. Bivariate Cox regression analysis was done to investigate the relationships between mortality and independent variables. Subsequently, to evaluate factors associated with in‐hospital mortality, a multivariate Cox regression analysis (reported with adjusted hazard ratios [AHRs] with 95% CI) was performed, including all independent variables with biological plausibility for in‐hospital mortality at a *p* value of 0.25 on bivariate Cox regression analysis. All *p* values calculated were two‐sided, and a *p* value less than 0.05 was used to declare statistical significance.

### 2.10 Term/operational definition

#### 2.10.1 Regular physical exercise

An individual's physical activity status before the current admission was evaluated by using the global physical activity questionnaire,^34^ and those who exercised for 30 min a day for 5 times a week were considered physically active.

#### 2.10.2 Smoking status^35^

A patient was classified as a “never smoker” if he or she had never smoked or had smoked <100 cigarettes in his or her lifetime but had quit smoking during the previous 28 days. While a patient who had smoked at least 100 cigarettes in their lives but had stopped smoking in the previous 28 days was considered an “ex‐smokers.” A patient was designated as a “current smoker” if he or she had smoked 100 cigarettes in his or her lifetime and had smoked in the previous 28 days.

## 3 RESULT

### 3.1 A summary of participants in the study

A sample of 167 patients with HE were screened for eligibility criteria, with 27 participants being reasonably excluded. Finally, 140 participants with HE were recruited for the study (Figure 1).

**Figure 1:** Chart showing patients with hypertensive emergency screened for eligibility and included in the study.

### 3.2 Sociodemographic and behavioral features of the participants in the study

The average age of the study participant was 52.79 ± 13.57 years. In terms of sex, the participants were predominantly males, 108 (77.1%). More than half, 84 (60.0%), of the participants were rural residents. The majority of the participant, 82(58.5%), reported regular physical exercise before the current admission. Self‐reported salt consumption was captured in 118 (84.3%) participants (Table 1).

**Table 1:** Sociodemographic and behavioral characteristics of participants with HE admitted to the emergency ward of JMC

Variables	Frequency (%)
Sex	
Male	108 (77.1)
Female	32 (22.9)
Age (years), mean ± SD	52.79 ± 13.57
Residence	
Urban	56 (40.0)
Rural	84 (60.0)
Marital status	
Single	9 (6.4)
Married	113 (80.7)
Divorced	1 (0.7)
Widow	17 (12.1)
Occupational status	
Housewife	23 (16.4)
Farmer	57 (40.7)
Merchant	25 (17.9)
Employed (Govt/NGO)	20 (14.3)
Retired	15 (10.7)
Educational status	
Cannot read or write	62 (44.3)
Primary school	45 (32.1)
Secondary school	11 (7.9)
Tertiary and above	22 (15.7)
Khat chewing	
Chewer	24 (17.1)
Previous chewer	63 (45.0)
Never	53 (37.9)
Smoking history	
Current smoker	15 (10.7)
Ex‐smoker	4 (2.9)
Nonsmoker	121 (86.4)
Alcohol drinking habit	25 (17.9)
Physical exercise before the current admission	82 (58.5)
Salt consumption	118 (84.3)

Abbreviations: Govt, Governmental Organization; HE, hypertensive emergency; JMC, Jimma Medical Center; NGO, nongovernmental organization; SD, standard deviation.

### 3.3 Clinical characteristics

The majority of the participants, 85 (60.7%), had a previously known hypertension and most of these participants, 68 (80.0%), had no regular follow‐up. Upon arrival at the emergency ward, the median (IQR) SBP and DBP of the study participants were 200 (190–211) and 115 (110–125) mmHg, respectively. Diabetes mellitus, 37 (27.6%), was the most common comorbid disease, followed by infectious diseases, 32 (23.9%). On the contrary, the most common clinical presentations upon arrival at the hospital were palpitation, 73 (52.1%), and vomiting, 67 (47.9%) (Table 2).

**Table 2:** Baseline clinical features of patients with HE admitted to the emergency ward of JMC

Variables	Frequency (%)
Hypertension diagnosis	
Known	85 (60.7)
New	55 (39.3)
Regular follow‐up (*n* = 85)	17 (20.0)
SBP (mmHg) at admission, median (IQR)	200 (190–211)
DBP (mmHg) at admission, median (IQR)	115 (110–125)
Family history of hypertension	16 (11.4)
Comorbidity	134 (95.7)
Specific comorbidity	
Diabetes mellitus	37 (27.6)
Infection	32 (23.9)
Chronic renal disease	34 (25.4)
Heart failure	12 (8.9)
Acute coronary syndrome	12 (8.9)
Ischemic heart disease	7 (5.2)
Clinical signs and symptoms on admission	
Palpitation	73 (52.1)
Vomiting	67 (47.9)
Shortens of breath	66 (47.1)
Nausea	65 (46.4)
Paralysis	64 (45.7)
Chest pain	48 (34.3)
Pain	43 (30.7)
Tachypnea	45 (32.1)
Headache	36 (25.7)
Vision changes	35 (25.0)
Aphasia	27 (19.3)
Hyperthermia	8 (5.7)

Abbreviations: DBP, diastolic blood pressure; HE, hypertensive emergency; IQR, interquartile range; JMC, Jimma Medical Center; SBP, systolic blood pressure.

The most common target organ complication noted were hemorrhagic stroke (38.0%) and acute kidney injury (27.1%) (Table 3).

**Table 3:** Target organ damages diagnosed in HE patients admitted to the emergency ward of JMC

Target organ damage	Frequency (%)
Hemorrhagic stroke	53 (38.0)
Acute renal failure	38 (27.1)
Ischemic stroke	14 (10.0)
Hypertensive retinopathy	12 (8.6)
Hypertensive encephalopathy	8 (5.7)
ST‐elevated myocardial infarction	8 (5.7)
Acute congestive heart failure	6 (4.3)
Aortic dissection	1 (0.7)

Abbreviations: HE, hypertensive emergency; JMC, Jimma Medical Center.

### 3.4 Medication profile of the participants

Before the current admission, more than half of the participants (55.0%) had stopped taking antihypertensive medications. During their hospitalization, a total of 430 medications were prescribed. Of the medications prescribed, hydralazine, 47 (33.6%), was the most frequent, followed by short‐acting nifedipine, 43 (30.7%), and captopril, 24 (17.1%) (Table 4).

**Table 4:** Antihypertensive drug use and related factors among hospitalized patients with HE at the emergency ward of JMC

Medication history		Frequency (%)
Past medication history		
Duration on antihypertensive medication (years), mean (±SD)		2.4 (±4.0)
Specific antihypertensive medications used		
Hydrochlorothiazide PO		27 (19.3)
Enalapril PO		21 (15.7)
Amlodipine PO		22 (15.7)
Atenolol PO		3 (2.1)
Discontinued antihypertensive medication(s) before the present admission		
Yes		77 (55.0)
No		63 (45.0)
Reason for stopping medication(s)		
Being asymptomatic		34 (24.3)
Forgetfulness		14 (10.0)
Affordability issue		29 (20.7)
Medication availability		63 (45.0)
Medications used to treat HE at the emergency ward		
Hydralazine IV		47 (33.6)
Short‐acting nifedipine PO		43 (30.7)
Captopril PO		24 (17.1)
Metoprolol tartrate PO/IV		22 (15.7)
Captopril PO and hydralazine IV		3 (2.1)
Captopril and nifedipine PO		1 (0.7)

Abbreviations: HE, hypertensive emergency; IV, intravenous; JMC, Jimma Medical Center; PO, by mouth.

### 3.5 In‐hospital outcomes of HE

The median (IQR) SBP and DBP blood pressure had fallen to 142 (136.25–150) and 90 (80–90) mmHg till discharge, respectively. A total of 16 (11.4%, 95% CI: 6.7–17.9) in‐hospital mortality were recorded. The overall mean (±SD) length of stay and the mean time to mortality at the hospital were 8.53 ± 3.61 and 2.88 ± 2.47 days, respectively (Table 5).

**Table 5:** Status of discharge, average blood pressure records on admission, and discharge in patients with HE admitted to the emergency ward of JMC

Patients with HE (*n* = 140)	Time at which average blood pressure was recorded			
	At admission			At discharge/death
Median SBP (IQR) (mmHg)	200 (190–211)			142 (136.25–150)
Median DBP (IQR) (mmHg)	115 (110–125)			90 (80–90)
Discharge status and duration of hospital stay				
Status discharge			
Alive		124 (88.6%)		
Death		16 (11.4%)		
Duration of hospital stay, in days (mean ± SD)		8.53 ± 3.61		
The average time to death, in days (mean ± SD)		2.88 ± 2.47		

Abbreviations: DBP, diastolic blood pressure; HE, hypertensive emergency; IQR, interquartile range; JMC, Jimma Medical Center; SBP, systolic blood pressure; SD, standard deviation.

As the hospital stay increased, the survival of patients not undergoing regular physical exercise before the current admission, that is, mean days of 14.35 (95% CI: 12.59–16.11) was less than those with undergoing regular physical exercise (i.e., mean days of 17.39; 95% CI: 16.71–18.06; log‐rank: *p* = 0.001) (Figure 2).

**Figure 2:** Kaplan–Meier survival analysis of patients admitted with HE over the length of their hospital stay was stratified by the behavior of regular physical exercise before the current admission. HE, hypertensive emergency.

### 3.6 Factors predicting in‐hospital mortality

Age (crude hazard ratio (CHR) = 1.051, 95% CI: 1.013–1.092, *p* = 0.009), regular physical exercise before the current admission (CHR = 6.65, 95% CI: 1.893–23.389, *p* = 0.003), discontinue antihypertensive medication (CHR = 3.720, 95% CI: 1.061–13.088, *p* = 0.040) were associated with in‐hospital mortality on bivariate Cox regression analysis. A total of eight variables were selected for multivariate Cox regression analysis, and not doing regular physical exercise before the current admission (AHR = 4.629, 95% CI: 1.171–18.294, *p* = 0.015) was significantly associated with in‐hospital mortality (Table 6).

**Table 6:** Cox regression analysis, both bivariate and multivariate, to determine factors linked with the discharge status in patients with HE at the emergency unit of JMC

Variable		Discharge status		Bivariate analysis		Multivariate analysis	
		Alive (*n* = 124) (%)	Death (*n* = 16) (%)	CHR (95%CI)	*p* Value	AHR [95% CI]	*p* Value
Age (years), mean ± SD		51.7 ± 12.7	61.2 ± 17.5	1.051 [1.013–1.092]	**0.009**	1.016 [0.969–1.065]	0.513
DBP, mean ± SD		118.5 ± 12.7	114.0 ± 14.1	0.97 [0.93–1.06]	0.196	0.979 [0.932–1.028]	0.394
Duration of hypertension, mean ± SD		2.18 ± 3.876	4.00 ± 4.487	1.082 [0.987–1.185]	0.093	0.963 [0.850–1.092]	0.560
Doing regular physical exercise before the current admission							
No		45 (36.3)	13 (81.3)	6.65 [1.893–23.389]	**0.003**	4.629 [1.171–18.294]	**0.015**
Yes		79 (63.7)	3 (18.8)	1		1	
Comorbidity							
Yes		78 (62.9)	14 (87.5)	3.843 [0.873–16.915]	0.075	1.731 [0.139–21.486]	0.670
No		46 (37.1)	2 (12.5)				
Knowing being hypertensive before the current admission							
No		54 (43.5)	3 (18.8)	0.326 [0.093–1.145]	0.080	1.343 [0.149–12.077]	0.792
Yes		70 (56.5)	13 (81.3)	1		1	
On admission shortness of breath							
Yes		56 (45.2)	10 (62.5)	1.875 [0.681–5.161]	0.224	1.375 [0.478–3.959]	0.555
No		68 (54.8)	6 (37.5)	1		1	
Discontinue antihypertensive medication							
Yes		65 (52.4)	13 (81.3)	3.720 [1.061–13.088]	**0.040**	1.900 [0.456–7.922]	0.378
No		59 (47.6)	3 (18.8)	1		1	

*Note*: Bold values indicate statistically significant association between outcome variable and independent variables.

Abbreviations: AHR, adjusted hazard ratio; CHR, crude hazard ratio; CI, confidence interval; DBP, diastolic blood pressure; HE, hypertensive emergency; IV, intravenous; JMC, Jimma Medical Center; SD, standard deviation; SBP, systolic blood pressure.

## 4 DISCUSSION

This prospectively conducted study included 140 HE patients to assess in‐hospital outcomes at JMC. Among the study participants, hemorrhagic stroke (38.0%) was the most frequent complication noted and in‐hospital mortality rate was recorded in 11.4% of them.

The finding of an 11.4% mortality rate in patients with HE in this study is nearly similar to a report from Gonder, northwest Ethiopia, 11.6%,^11^ France, 12.5%,^36^ Italy, 14.5%,^37^ and Greece, 14.7%.^38^ However, the higher mortality rate was reported in Nigeria, 22.1%^39^ and 42.9%,^12^ Tanzania, 26.8%,^40^ Democratic Republic of Congo (DRC), 22.2%,^41^ and Addis Ababa, Ethiopia, 16.9%.^26^ This difference might be justified by most of the previous studies^12^, ^39^, ^41^ that was conducted a decade ago since the management of complicated hypertension advances across years both in the diagnostic and therapeutic approaches and results in an improvement in patient outcomes.^42^ Furthermore, methodological heterogeneity may have a share in this variation.

In the present study, the median SBP and DBP have fallen from 200–142 to 115–90 mmHg at discharge, respectively, which is slightly different from a report from Gonder, northwest Ethiopia (58 vs. 50 mmHg reduction in SBP and 25 vs. 20 mmHg reduction in DBP).^11^ This discrepancy could be because the previous study retrieved data from the patient chart, while in the current study, blood pressure was directly measured and recorded from the patient.

In this study, the most common clinical manifestation of patients presented with HE was palpitation (52.1%), followed by vomiting (47.9%), shortness of breath (47.1%), and paralysis (45.7%). A comparable result was reported from DRC,^43^ Pakistan,^44^ and Gonder, Ethiopia.^11^

Many of the previous studies revealed that brain‐related events, mainly hemorrhage and ischemic stroke, are the most common complications of HE.^22^, ^26^, ^43^, ^45^, ^46^, ^47^ Similarly, stroke accounted for 48.0% (38.0% hemorrhagic stroke and 10.0% ischemic stroke) of the complications recorded among HE patients in the current study.

In our study, the average (±SD) number of days spent in the hospital was 8.53 ± 3.61, which is higher than a study from Pakistan, 2.46 (±0.164) days.^44^ However, this finding is lower than a report from the United States of America, 11.7 days,^48^ DRC, 11.4 ± 5.5 days,^49^ and Addis Ababa, Ethiopia, 11.45 (±11.48) days.^26^ This discrepancy might be because of differences in quality of care, advancement in treatment protocol across years, and heterogeneity of the study population.

Antihypertensive medications used to treat HE were varied across studies and inconsistent with the European Society of Cardiology and the 2020 International Society of Hypertension practice guidelines recommendation: labetalol or nicardipine as the first‐line medications used to treat HE.^18^, ^19^ A report from Thailand revealed that hydralazine was a frequently prescribed agent for the management of HE,^50^ which is similar to the current finding, where hydralazine was prescribed and used in 33.6% of the patient management. Unlike the current study, a report from Gonder, Ethiopia showed that captopril (45.3%), followed by hydralazine (36%), were the most commonly used agents.^11^, ^51^ These might be because of differences in the availability of medications across study settings.

Plenty of evidence revealed the exponential relationship between mortality and age.^52^, ^53^, ^54^ In the present study, age was significantly associated with all‐cause in‐hospital mortality on bivariate Cox regression analysis, but the association was lost after adjustment with other covariates in multivariate Cox regression analysis. In fact, aging causes the accumulation of damaged and deteriorated cells, tissues, and organs, which eventually end in mortality. Similarly, previous studies revealed the protective associations of baseline physical activity against mortality from cardiovascular disease.^55^, ^56^, ^57^ A consistent result was reported in the current study; patients not doing regular physical exercise before the current admission increase the risk of in‐hospital mortality by more than fourfold.

To the best of our knowledge, this is the first study to report HE admission outcomes and predictors at JMC. Despite all its merits, the current study has some limitations. Important factors like the lipid profile, coagulation profile, and consciousness level upon admission that may affect the outcome of HE are not well examined. The consideration of a single setting and the current study's small sample could limit the findings' generalizability. Additionally, the study did not address the long‐term outcomes of HE.

## 5 CONCLUSION

In summary, about one‐tenth of those with HE died in this study. The frequent HE complications were hemorrhagic stroke and acute renal damage. Patients with HE who did not engage in regular physical activity before their current hospitalization are more likely to die. The authors recommend that healthcare professionals and other concerned bodies have to strengthen patient education and encourage patients to integrate regular physical exercise with daily activities.

## AUTHOR CONTRIBUTIONS

**Mengist Awoke Yizengaw**: Conceptualization; data curation; formal analysis; methodology; project administration; validation; writing – original draft; writing – review and editing. **Kisi Chemeda**: Conceptualization; data curation; formal analysis; funding acquisition; investigation; methodology; project administration; supervision; visualization; writing – original draft; writing – review and editing. **Kabaye Kumela**: Conceptualization; data curation; formal analysis; methodology; supervision; validation; visualization; writing – original draft; writing – review and editing. **Behailu Terefe Tesfaye**: Conceptualization; data curation; formal analysis; investigation; methodology; supervision; validation; visualization; writing – original draft; writing – review and editing.

## CONFLICT OF INTEREST

The authors declare no conflict of interest.

## TRANSPARENCY STATEMENT

The lead author Mengist Awoke Yizengaw affirms that this manuscript is an honest, accurate, and transparent account of the study being reported; that no important aspects of the study have been omitted; and that any discrepancies from the study as planned (and, if relevant, registered) have been explained.

## ETHICS STATEMENT

The Institutional Review Board (IRB) of Jimma University provided permission to conduct the study and clearance under the reference number IRB 00019/2020 and all methods were conducted as per the principles of the Declaration of Helsinki. Before data collection began, the patient signed a written informed permission form.

## Data Availability

On reasonable request, the corresponding author will provide the data sets created and/or analyzed during the current work.
